This article has been retracted.

# Clinicopathological Features of 166 Cases of Invasive Ductal Breast Carcinoma and Effect of Primary Tumor Location on Prognosis after Modified Radical Mastectomy

**DOI:** 10.1155/2022/3158956

**Published:** 2022-06-18

**Authors:** Shiman Chen, Liang Yang, Yaqiong Li

**Affiliations:** Department of Thyroid and Breast and Vascular Surgery, Renmin Hospital, Hubei University of Medicine, Shiyan, Hubei 442000, China

## Abstract

**Objective:**

To investigate the clinicopathological features of 166 cases of invasive ductal carcinoma (IDC) of the breast and to analyze the effect of the location of the primary tumor on the prognosis of modified radical mastectomy.

**Materials and Methods:**

The clinical data of 166 patients with IDC who underwent modified radical mastectomy in our hospital from May 2015 to May 2017 were retrospectively analyzed. The clinicopathological features of IDC patients were recorded. Univariate analysis and the multivariate logistic regression model were used to analyze the relationship between the location of the primary tumor and the prognosis of IDC patients after modified radical surgery. The effect of primary tumor location on the prognosis of modified radical resection was used with Survival curve analysis.

**Results:**

Among the patients in the central region, 13.33% had tumors >5 cm in diameter, which was higher than those in the other four groups. Among the patients in the upper inner quadrant, 59.38% received hormone therapy after operation, which was higher than those in the other four groups (*P* < 0.05). There were no significant differences in age, menopause, histological grading, molecular typing, lymph node metastasis, vascular invasion, radiation therapy, and chemotherapy among different groups (*P* > 0.05). Univariate analysis showed that molecular typing, lymph node metastasis, vascular invasion, and location of the primary tumor were all related to the prognosis of IDC patients after modified radical surgery, and the differences were statistically significant (*P* < 0.05). Logistic regression analysis showed that molecular typing, lymph node metastasis, vascular invasion, and primary tumor location were all independent influencing factors for prognosis of IDC patients after modified radical surgery (*P* < 0.05). As of 31 May 2021, there were 11 patients with recurrence and metastasis and 20 patients with death. The median survival time in the outer upper quadrant group was 80 months, which was higher than that in the outer lower quadrant group by 72 months, the median survival time in the central region group by 71 months, the median survival time in the inner upper quadrant group by 67 months, and the median survival time in the inner lower quadrant group by 61 months. The log-rank test showed all *P* < 0.001.

**Conclusion:**

Patients with primary tumors located in the central area have larger tumor diameters. Patients located in the central area, upper inner quadrant, and lower inner quadrant are more likely to have lymphatic metastasis, have a more serious condition, and have a shorter prognosis survival time. Unluminal type, multiple lymph node metastases, vascular invasion, and the location of the primary tumor in the inner quadrant are all independent risk factors for prognosis in patients after modified radical surgery for IDC.

## 1. Introduction

Breast cancer is one of the most common malignancies in women. In recent years, its incidence has been increasing year by year in the global scope. Invasive ductal carcinoma (IDC) of the breast is the most common type of breast cancer and belongs to nonspecific invasive carcinoma of the breast. Clinically, patients often have breast lumps and nipple discharge [1, 2]. IDC often affects the physical and psychological health of women due to the younger onset group, the tendency of lymphatic metastasis and recurrence in advanced patients, and the influence on the appearance of breasts after surgical resection [3, 4]. Therefore, early diagnosis and treatment of IDC are extremely important.

At present, the treatment methods for IDC mainly include radical surgery, modified radical surgery, and postoperative chemoradiotherapy [5, 6]. Among them, modified radical surgery is an effective method for the treatment of IDC. It can preserve the pectoralis minor and pectoralis major muscles of the affected side of the patient and minimize the damage to the shape of the breast. Compared with traditional surgery, modified radical surgery not only ensures the thoroughness of tumor resection but also satisfies the pursuit of beauty for female patients. It is the most commonly used surgical method in clinical practice at present. [7, 8]. With the nipple as the center, the breast can be divided into five positions, including four quadrants and a central area. The primary tumor is located in different locations, and the progression speed of the disease is also different. In this study, we retrospectively analyzed the follow-up data of 166 IDC patients within five years after modified radical surgery, summarized the clinicopathologic features of these patients, and analyzed the impact of the location of primary tumors on the prognosis of modified radical surgery. The specific report is as follows.

## 2. Information and Methods

### 2.1. General Information

A total of 166 IDC patients undergoing modified radical mastectomy in our hospital from May 2015 to May 2017 were retrospectively collected. Their age ranged from 25 to 75 years old, with an average of 50.79 ± 9.61 years old.

### 2.2. Inclusion Criteria

Inclusion criteria were as follows: (1) Meets breast cancer IDC diagnostic criteria; (2) the pathological diagnosis is unilateral IDC; (3) receiving modified radical mastectomy; (4) having complete clinical and pathological data and follow-up information.

### 2.3. Exclusion Criteria

Exclusion criteria were as follows: (1) Preoperative neoadjuvant chemotherapy; (2) distant metastasis has occurred at the time of initial treatment; (3) the location of the tumor is located in the boundary area of each quadrant; (4) multifocal breast cancer; (5) male breast cancer.

### 2.4. Primary Tumor Location

Tumor location was determined on the basis of a preoperative imaging report (color Doppler ultrasound, mammography, or MRI) closest to the date of surgery and intraoperative measurements. A horizontal and vertical line was drawn with the nipple as the center, which divided the breast into outer upper, outer lower, inner upper, and inner lower. The nipple and areola were the central area, 5 regions in total. The location of the primary tumor was divided into the outer upper quadrant, the outer lower quadrant, the inner upper quadrant, the inner lower quadrant, and the central region, which included the nipples and areola complex.

### 2.5. Postoperative Follow-Up

A follow-up was performed every 3 months for the 2-year postoperative period, semiannually from the 3rd year, and annually after the 5th year. The follow-up included breast tumor markers, breast ultrasound, mammography chest X-rays and abdominal ultrasound, and CT and whole-body bone scans when necessary. The follow-up deadline of all patients was May 31, 2021. If a patient had tumor recurrence, metastasis, or death, the follow-up would be deemed as terminated. The median follow-up time was 73 months. During the follow-up period, there were 11 patients with recurrence and metastasis and 20 patients with death. The clinical and pathological characteristics such as age, menopause or not, tumor diameter, histological grade, molecular classification, lymph node metastasis, vascular invasion, radiotherapy, chemotherapy, endocrine therapy, and the location of the primary tumor were recorded.

### 2.6. Statistical Processing

Data processing was performed using SPSS22.0 software. The enumeration data were expressed as %, and the comparison was performed using the *χ*2 test. The multivariate logistic regression model was used for multivariate analysis. Kaplan–Meier survival curve was used to analyze the relationship between the location of the primary tumor and the prognosis of modified radical mastectomy. The log-rank test was used for comparison. The test level was *α* = 0.05, and *P* < 0.05 indicated that the difference was statistically significant.

## 3. Results

### 3.1. Clinical Pathological Features of IDC

Among the patients in the central region, 13.33% (2/15) had tumors >5 cm in diameter, which was higher than those in the other four groups. Among the patients in the upper inner quadrant, 59.38% (19/32) received hormone therapy postoperatively, which was higher than those in the other four groups (*P* < 0.05). There were no significant differences in age, menopause, histological grading, molecular classification, lymph node metastasis, vascular invasion, radiation therapy, and chemotherapy among different groups (*P* > 0.05) (see Table 1).

### 3.2. Univariate Analysis of Prognosis of IDC Patients after Modified Radical Mastectomy

Univariate analysis showed that molecular typing, lymph node metastasis, vascular invasion, and location of the primary tumor were all related to the prognosis of IDC patients after modified radical mastectomy, and the differences were statistically significant (*P* < 0.05) (see Table 2).

### 3.3. Multivariate Logistic Regression Analysis on Prognosis of IDC Patients after Modified Radical Mastectomy

Multivariate logistic regression analysis showed that molecular typing, lymph node metastasis, vascular invasion, and primary tumor location were all independent risk factors for prognosis of IDC patients after modified radical mastectomy (*P* < 0.05) (see Tables 3 and 4).

### 3.4. The Prognostic Effect of Different Tumor Locations on IDC Patients after Modified Radical Surgery

As of 31 May 2021, there were 11 patients with recurrence and metastasis and 20 patients with death. The median survival time in the outer upper quadrant group was 80 months, which was higher than that in the outer lower quadrant group by 72 months, the median survival time in the central region group by 71 months, the median survival time in the inner upper quadrant group by 67 months, and the median survival time in the inner lower quadrant group by 61 months. The log-rank test showed all *P* < 0.001 (see Figure 1).

## 4. Discussion

Invasive breast cancer is a common type in breast cancer patients, and IDC is in the majority. IDC accounts for 70%–80% of invasive breast cancer, and patients are often accompanied by breast masses, pitting nipples, and other clinical manifestations [9, 10]. At present, the main examination methods of IDC include mammography, color Doppler ultrasound, CT, and MRI [11, 12]. The primary tumor is located in different locations and lymph node metastasis occurs at different rates. For early IDC patients with tumor diameter <3 cm and no axillary lymph node metastasis or only slight metastasis and no distant metastasis, the therapeutic effect is good, and more than 90% of patients can be cured for a long time [13, 14]. However, early IDC patients did not have typical clinical symptoms and signs, and it was difficult to detect them during normal times. The diagnosis needed to be made based on imaging and pathology examinations, which easily missed the optimal treatment period and posed a serious threat to women's health [15, 16]. Therefore, early diagnosis and treatment of IDC are very important.

Among the patients in the central region, 13.33% (2/15) had tumors >5 cm in diameter, which was higher than those in the other four groups. Among the patients in the upper inner quadrant, 59.38% (19/32) received endocrine therapy after operation, which was higher than that in the other four groups. There were no significant differences in age, menopause or not, histological grade, molecular classification, lymph node metastasis, vascular invasion, radiotherapy, and chemotherapy of patients among different groups. The reason for this was analyzed as the existence of a nipple-areolar complex in the central area made it difficult to detect the primary tumor, resulting in a larger tumor volume for the first detection. After the operation, the patient needs postoperative radiotherapy and chemotherapy to prevent further development of the disease [17]. Lymph node metastasis is more likely to occur in tumors in the upper inner quadrant, and endocrine therapy can improve endocrine function of patients, thereby avoiding the growth and metastasis of cancer cells in patients [18, 19].

Our results show that un-luminal type, multiple lymph node metastases, vascular invasion, and the location of the primary tumor in the inner quadrant are all independent risk factors for the prognosis of IDC patients after modified radical surgery. The reason was analyzed as follows: IDC is a highly heterogeneous tumor, different molecular types of IDC have different biological characteristics, prognosis, and sensitivity to treatment, which affect the prognosis of patients after modified radical surgery [20, 21]. The more lymph node metastasis is, the more serious the vascular invasion, which often indicates the hematogenous metastasis and lymphatic metastasis of the tumor. Therefore, the more serious the disease is, which is not conducive to the prognosis of the patient [22]. Unluminal type includes Her-2 overexpression type and triple-negative breast cancer. Although these two types are sensitive to chemotherapy, they have been found in clinical practice to have a poorer prognosis than the luminal type, which has been widely recognized in clinical practice. Lymphatic metastasis is the most common metastasis mode of IDC. The prognosis of IDC patients with primary tumors located in the central area, upper inner quadrant, and lower inner quadrant is significantly worse than those of patients in the upper outer quadrant and lower outer quadrant. There are rich lymphatic vessels at the nipples in the central area, and the cancer cells located in the central area are easy to undergo lymphatic metastasis through the rich lymphatic vessels around, which are the independent risk factors for patients with IDC after modified radical surgery [23, 24]. The internal mammary gland is the second largest lymphatic metastasis pathway after the axillary lymph node. For IDC patients with primary tumors located in the upper inner quadrant, lower inner quadrant, and central region, the tumor was closer to the internal mammary gland lymphatic drainage pathway, and it was more prone to lymphatic metastasis, which was not conducive to the prognosis of patients [25]. In addition, internal mammary lymph nodes are characterized by deep anatomical location and small size, which are difficult to be detected clearly by mammography and color Doppler ultrasound, thus delaying the treatment time and unfavorable to the prognosis [26].

As of 31 May 2021, the median survival time in the outer upper quadrant group was 80 months, which was higher than that in the outer lower quadrant group by 72 months, the median survival time in the central region group by 71 months, the median survival time in the inner upper quadrant group by 67 months, and the median survival time in the inner lower quadrant group by 61 months. The reason was analyzed as follows: lymphatic metastasis is the most important mode of metastasis of IDC tumors. The closer the primary tumor is to the internal mammary lymphatic metastasis pathway, the more likely the cancer cells will develop lymphatic metastasis and the severer the disease will be, which will affect the prognosis of patients undergoing modified radical mastectomy [27]. As a result, the five-year survival rate of IDC patients will be reduced, and the five-year survival rate of patients with primary tumors located in the central area, the inner upper quadrant, and inner lower quadrant will be lower than that of patients located in the outer upper quadrant and outer lower quadrant. In addition, due to the excessive penetration of mammography to the nipple-areolar complex, tumors in the central region are often overlooked, requiring the combination of multiple imaging techniques [28]. The molybdenum target detection rate of breast cancer in the central region is low, and the tumor is detected in a late stage, which delays the treatment time and reduces the five-year survival rate of patients [29].

In conclusion, patients with primary tumors located in the central area have larger tumor diameters. Patients located in the central area, upper inner quadrant, and lower inner quadrant are more likely to have lymphatic metastasis, have a more serious condition, and have a shorter prognosis survival time. They are the independent risk factors for prognosis after modified radical surgery. A good understanding of IDC and timely diagnosis and treatment can effectively improve the prognosis and increase the five-year survival rate of patients.

## Figures and Tables

**Figure 1:** Prognostic survival curves of IDC patients with different tumor locations after modified radical mastectomy.

**Table 1:** Clinical pathological features of IDC.

Clinical pathological features		Cases (*n* = 166)	Outer upper quadrant (*n* = 94)	Outer lower quadrant (*n* = 17)	Central area (*n* = 15)	Inner upper quadrant (*n* = 32)	Inner lower quadrant (*n* = 8)	*χ* ^*2*^ value	*P*
Age (years)	<35	8	5	1	0	2	0	0.194	0.986
	≥35 and <50	72	39	7	7	13	6		
	≥50	86	50	9	8	17	2		
Menopause	No	89	50	10	8	17	4	0.983	0.979
	Yes	77	44	7	7	15	4		
Tumor diameter (cm)	≤2	43	17	8	3	12	3	17.114	0.009
	>2且≤5	118	75	9	10	19	5		
	>5	5	2	0	2	1	0		
Histological grading	Type I	7	4	1	0	0	2	4.950	0.550
	Type II	95	58	7	9	18	3		
	Type III	64	32	9	6	14	3		
Molecular typing	Luminal A	24	13	3	3	4	1	2.103	0.607
	Luminal B	81	46	9	7	17	2		
	Triple negative	41	23	5	5	5	3		
	Her-2 (+)	20	12	0	0	6	2		
Lymph node metastasis	No	97	52	10	9	20	6	3.560	0.101
	1∼3 nodes	41	23	3	5	8	2		
	≥4 nodes	28	19	4	1	4	0		
Vascular infiltration	No	162	93	16	14	31	8	2.679	0.444
	Yes	4	1	1	1	1	0		
Radiation therapy	No	111	61	12	10	21	7	0.213	0.975
	Yes	55	33	5	5	11	1		
Chemotherapy	No	26	14	4	2	6	0	0.515	0.798
	Yes	140	80	13	13	26	8		
Hormone therapy	No	76	38	8	11	13	6	8.771	0.032
	Yes	90	56	9	4	19	2		

**Table 2:** Univariate analysis of prognosis of IDC patients after modified radical mastectomy (*n*, %).

Clinicopathologic features		Cases (*n* = 166)	5-year survival rate	*χ* ^*2*^ value	*P* value
Age (years)	<35	8	75.00% (6/8)	4.803	0.091
	≥35 and <50	72	83.33% (60/72)		
	≥50	86	93.02% (80/86)		
Menopause	No	89	87.64% (78/89)	0.018	0.895
	Yes	77	88.31% (68/77)		
Tumor diameter (cm)	≤2	43	93.02% (40/43)	1.596	0.450
	>2 and ≤5	118	86.44% (102/118)		
	>5	5	80.00% (4/5)		
Histological grading	Type I	7	100% (7/7)	0.792	0.782
	Type II	95	94.74% (90/95)		
	Type III	64	93.75% (60/64)		
Molecular typing	Luminal type	105	92.38% (97/105)	5.290	0.021
	Unluminal type	61	80.33% (49/61)		
Lymph node metastasis	No	97	93.81% (91/97)	8.556	0.000
	1∼3 nodes	41	82.92% (34/41)		
	≥4 nodes	28	75.00% (21/28)		
Vascular infiltration	No	162	88.89% (144/162)	5.472	0.025
	Yes	4	50.00% (2/4)		
Radiation therapy	No	111	84.68% (94/111)	3.375	0.066
	Yes	55	94.55% (52/55)		
Chemotherapy	No	26	80.77% (21/26)	1.501	0.221
	Yes	140	89.29% (125/140)		
Hormone therapy	No	76	82.89% (63/76)	3.383	0.066
	Yes	90	92.22% (83/90)		
Primary tumor location	Outer upper quadrant	94	94.47% (89/94)	12.720	0.000
	Outer lower quadrant	17	88.24% (15/17)		
	Central area	15	80.00% (12/15)		
	Inner upper quadrant	32	78.13% (25/32)		
	Inner lower quadrant	8	62.50% (5/8)		

**Table 3:** Assignment for multivariate analysis of factors.

Influencing factors	Assignment
Molecular typing	Luminal type = “0”; unluminal type = “1”
Lymph node metastasis	No = “0”, 1∼3 nodes = “1”, ≥4 nodes = “2”
Vascular infiltration	No = “0”, yes = “1”
Primary tumor location	Outer upper quadrant = “0,” outer lower quadrant = “1,” central area = “2,” inner upper quadrant = “3,” inner lower quadrant = “4”

**Table 4:** Multivariate logistic regression analysis on prognosis of IDC patients after modified radical mastectomy.

Variable	*B*	Wald's	OR	95% CI	*P*
Molecular typing	0.699	3.028	1.115	1.142∼1.825	0.044
Lymph node metastasis	0.758	2.226	1.652	1.315∼1.998	0.032
Vascular infiltration	0.652	2.958	1.369	1.109∼1.751	0.028
Primary tumor location	0.145	3.268	1.669	1.175∼1.987	0.011

## Data Availability

The datasets used and/or analyzed in the current study are available from the corresponding author upon request.
